# PEComa of the mesentery coexisting with colon cancer: a case report

**DOI:** 10.1186/s13000-015-0265-5

**Published:** 2015-04-18

**Authors:** Jarosław Wejman, Krzysztof Nowak, Lena Gielniewska, Magdalena Komorowska, Wojciech Dąbrowski

**Affiliations:** Department of Pathology, Professor Witold Orlowski Public Clinical Hospital, Medical Center for Postgraduate Education, Czerniakowska 231, 00-416 Warsaw, Poland; Department of General and Hematological Surgery, Institute of Hematology and Transfusion Medicine, Indiry Gandhi 14 street, 02-776 Warsaw, Poland

**Keywords:** PEComa, Mesentery tumor, Perivascular epithelioid cell, Mesenteric PEComa, PEC

## Abstract

Perivascular epithelioid cell tumor (PEComa) is a rare entity originating from mesenchymal tissue, which stains for both melanocytic and smooth muscle markers. We would like to present an unusual case of the PEComa of the mesentery which was unexpected discovery in a female patient with colonic adenocarcinoma. The tumour was revealed on the computer tomography and then resected during surgery, with subsequent chemotherapy for the colon adenocarcinoma. Furthermore we would like to discuss PEComa biology, emphasizing histological criteria of malignancy, possible treatment options and differential diagnosis which is mostly based on immunohistochemistry.

**Virtual slides: **The virtual slide(s) for this article can be found here: http://www.diagnosticpathology.diagnomx.eu/vs/1809062291157051.

## Background

According to WHO definition perivascular epithelioid cell tumor is a “mesenchymal tumor composed of histologically and immunohistochemically distinctive perivascular epithelioid cells” [1].The PEComa cell does not have a known “normal” counterpart and this tumor is characterized by expression both melanocytic (such as HMB-45) and smooth muscle markers (such as SMA). We would like to present a case of PEComa of the mesentery coexisting with colon adenocarcinoma. PEC tumors of mesentery are extremely rare entities, with only seven cases reported up to 2013y [2-5].

## Case presentation

The patient was a 67 years old female with symptoms of a partial bowel obstruction. On the CT scans there was concentric thickening of the colon wall 11–12 centimeters long. There was also a smooth, solid lesion measuring 2,8 × 3,1 × 3 cm in the mesentery, with a strong, homogenous contrast enhancement in the arterial phase (Figure 1). During the operation the rectum was also partially resected due to suspicion for cancer implants in the mucosa. After surgery she is treated with chemotherapy.

**Figure 1:** A CT showing tumour of the mesentery with prominent contrast enhancement.

Routine H&E stains were performed and immunohistochemical studies were done on the formalin- fixed, paraffin- embedded tissue sections using a panel of the following antibodies: CD10 clone 56C6, CD34 clone QBEnd 10, polyclonal rabbit anti- human CD 117(c-kit), polyclonal rabbit S-100, SMA 1A4 clone, HMB-45 clone HMB-45 and Vimentin clone V9, all antibodies provided by Dako.

Upon macroscopic examination of the received 20 cm of rectum and sigmoid there was a white, friable, tumor involving about 80% of the bowel wall perimeter measuring 5 cm and placed 2,5 cm from distal margin. There was a broad, deep infiltration of the mesorectum with a radial margin 0,1 cm. There was also a tissue fragment sent in an another container labeled as a lesion of mesentery measured 3,5 cm, which was white with a greyish center on the cross sections.

Histologically the tumor of the colon appeared as a moderately differentiated adenocarcinoma with broad involvement of underlying adipose tissue, with vast embolization of the lymphatic vessels of the bowel wall. There were cancer metastases in 7 out of 16 lymph nodes found. The cancer resection was not radical, with cancer foci in mucosa and submucosa in the distal margin.

The tumor of mesentery was composed of bundles of spindle cells with abundant cytoplasm, oval, blunt- shaped nuclei with inconspicuous nucleoli (Figures 2, 3), epithelioid foci were also present (Figure 4) Tumor was well- circumscribed, radically resected. There was no necrosis, mild atypia and mitotic activity 1-2/50 High Power Fields. Performed immunohistochemical studies showed strong reactivity for smooth muscle actin (SMA) within 100% of the tumor cells (Figure 5), reactivity for HMB-45 (within 30-40% of the tumor cells (Figure 6) and vimentin. Other immunohistochemical staining, such as desmin, CD 117, CD 10, AE1/AE3, S100 and CD34 showed to be negative. The tumor was diagnosed as a PEComa of the mesentery. No PEComa’s metastases to regional lymph nodes were found.

**Figure 2:** Spindle shaped PEC cells arranged in bundles, with no necrosis or vascular invasion; HE staining, magnification ×40.

**Figure 3:** Cytologic details od PEC spindle- shaped cells with mild atypia; HE staining, magnification ×40.

**Figure 4:** Focus of an epithelioid cells, cells with abundant cytoplasm, round nuclei and inconspicuous nucleoli are present; HE staining.

**Figure 5:** Strong cytoplasmatic reaction for SMA; magnification ×10.

**Figure 6:** Positive reaction for HMB-45 in about 30-40% of the tumour’s cells, magnification ×10.

## Conclusions

PEComas are group of tumors that are characterized by periepithelioid cell differentiation. Although until recently, such cell does not have a known physiological counterpart, it presents with peculiar immunochemical stainings for both melanocytic and smooth muscle markers [6,7]. In spite of its unclear histogenesis it is generally accepted entity now including angiomyolipoma of the kidney (AML), clear cell “sugar” tumor of the lung and lymphangioleiomyomatosis (LAM) as well as many other tumors previously classified mostly as low- grade sarcomas [8].

PEComas, other than mentioned above, arise mostly in the uterus and gastrointestinal tract. There is striking female to male predominance 4:1, even if female genital organs are excluded from these statistics. Up to 2013y, there was only seven reports of PEComa involving the mesentery [2-5]. The differential diagnosis in our case included leiomyosarcoma, epithelioid type of gastrointestinal stromal tumor (GIST) and alveolar soft part sarcoma. In our case differentiation between GIST, leiomyosarcoma and PEComa was based on immunohistochemical ground with CD117, CD34 showing negative results and positive HMB-45. Alveolar soft part sarcoma was excluded due to both morphological (delicate, vascular stroma in PEComa in contrast to dense, fibrous stroma in ASPS) and immunohistochemical features (HMB-45 and SMA stains negative in alveolar sarcoma).

After diagnosis it was necessary to estimate neoplasm’s biological potential. PEComa is a tumor of uncertain malignant potential There are no clear criteria for malignancy due to its rarity, but most authors agree that tumor size >5 cm, necrosis, infiltrative growth pattern, marked nuclear atypia, cellularity and high mitotic activity > 1/50 HPF increase the risk of malignant behavior [3,9]. There are no strict criteria yet to distinguish between benign tumour, tumor of uncertain malignant potential and malignant PEComa. However in presented case only one criterion- mitotic activity can indicate potentially malignant behavior, although two or more criteria histologically are believed to indicate malignancy [4]. However, other authors suggest that criteria of malignancy are: mitotic activity higher than 1/10 HPF and/or coagulative necrosis, whereas others mentioned above can label the neoplasm no more than uncertain malignant potential. Recently, new molecular and cytogenetic markers emerged, such as TFE3 gene translocation and X chromosome polysomy. TFE3 gene translocation probably correlate both with histologic appearance, such as more epithelioid look, rich vascularity, scanty adipose tissue and strong immunoreactivity for TFE3 protein as well as with clinical features: strong predilection for women, disease onset at younger age and absence of tuberous sclerosis in the background of the tumour genesis. However further studies are still indispensable, the differences mentioned above led some authors to distinguish tumors with TFE3 gene translocation as a distinct subtype of PEComa [10].

As a very rare neoplasm, the efficiency of therapies still are to be established, Most common approach is surgical removal of the tumor and “watchful waiting” strategy, but adjuvant radiotherapy and chemotherapy sometimes are being used [2,4,11].

In our case after surgery and histopathologic examination of the removed tissues patient is being treated with chemotherapy due to colon adenocarcinoma, with a “watchful waiting” approach to the PEComa, which can be justified in context of above.

## Consent

Written informed consent was obtained from the patient for publication of this Case Report and any accompanying images. A copy of the written consent is available for review by the Editor-in-Chief of this journal.

## Abbreviations

PEComa: Perivascular epithelioid cell tumor
H&E: Hematoxylin and eosin
CD: Cluster of differentiation
HMB-45: Human melanoma black 45
SMA: Smooth muscle actin
CT: Computed tomography
AML: Angiomyolipoma
LAM: Lymphangioleiomyomatosis
ASPS: Alveolar soft part sarcoma
GIST: Gastrointestinal stromal tumor
